RETRACTED

# Change in Health-Related Quality of Life in Cochlear Implant Recipients in China

**DOI:** 10.1155/2022/1770580

**Published:** 2022-03-26

**Authors:** Wenwen Zheng, Wei Cao, Shanwen Chen, Yifan Li, Yang Wang, Kun Yao, Jianxin Qiu

**Affiliations:** ^1^Department of Otolaryngology Head and Neck Surgery, The First Affiliated Hospital of Anhui Medical University, Hefei 230032, China; ^2^Department of Otolaryngology Head and Neck Surgery, The Affiliated Hefei Hospital of Anhui Medical University, Hefei 230011, China; ^3^Department of Otolaryngology Head and Neck Surgery, The Second Affiliated Hospital of Anhui Medical University, Hefei 230601, China; ^4^Department of Otorhinolaryngology-Head and Neck Surgery, Fuyang Hospital of Anhui Medical University, Fuyang 236112, China

## Abstract

**Objective:**

The objective is to assess the benefit of cochlear implants in health-related quality of life among postlingually deaf adults in China.

**Methods:**

Seventy-one postlingually deaf adult cochlear implant users in one cochlear implant center in China participated in this study. The HUI3 questionnaire as a measurement evaluated their quality of life. A cross-sectional analysis was conducted.

**Results:**

Cochlear implant had made statistically significant improvements in quality of life among postlingually deaf adults. The HUI3 scores were significantly better in four attributes (hearing, speech, emotion, and pain) after a cochlear implant. A positive correlation between change in hearing and improvement in emotion was significant. The change in pain and improvement in emotion also had a positive correlation. The duration of HA and CI use had no impact on the gain in HUI3 scores, and the baseline of hearing and emotion state had an influence on HUI3 gain.

**Conclusion:**

This study found cochlear implant users had a greatly improved hearing, speech, emotion, and pain, which made statistically significant improvement in quality of life among postlingually deaf adults. There was a statistically significant association between the change of emotion state and improvement in hearing level. We also found a statistically significant correlation between the reduction of feeling in pain and improvement in emotion. The change of quality of life seemed to be influenced by the primary state of emotion and hearing. We believe the measurement HUI3 is suitable for these patients in China.

## 1. Introduction

In China, by 2014, deaf adults only occupy 15% of the total cochlear implants (CI), although the population of adult hearing loss is more than 10 times of the number of pediatric hearing loss. Since national programs like China Disabled Persons' Federation (CDPF) were initiated, more and more adults have restored their hearing by CI [1]. To evaluate the benefit of CI, previous studies focused on the direct influence on hearing and speech improvement. Apart from these abilities, the CI could have an impact on other dimensions of life as well, for instance, social relations, emotion, and communications [2, 3]. Therefore, the evaluation of the influence of CI on patients' life requires an effective tool. The health-related quality of life (HRQOL) has been introduced to evaluate the influence of different interventions on people's daily life. There are many measurements available to assess the HRQOL of patients. These measurements comprehensively evaluate a patient's life from physical, social, and psychosocial aspects. These measurements include the generic World Health Organization Quality of Life (WHOQOL-BREF), Nijmegen cochlear implant questionnaire (NCIQ), EuroQol 5 dimensions (EQ-5D), Health Utility Index 3 (HUI3), and short-form 6 dimensions (SF-6D). Different measurements may get different results of the same medical treatment. Now, HUI3 is the most sensitive one to evaluate the QOL of patients with CI [4, 5]. Not only because HUI3 contains eight attributes, including hearing, but also HUI3 scores can be converted to a health utility, which is essential in cost-effectiveness analysis. The EQ-5D and SF-6D do not evaluate the hearing ability of the patient, and the others are unable to be converted to a utility score. The purpose of this study was to assess the effect of CIs using HUI3 measurement on postlingually deaf adults in China.

RETRACTED

## 2. Methods

A cross-sectional study was performed at the First Affiliated Hospital of Anhui Medical University, Anhui, China. This study was approved by the Health Research Ethics Committee. All subjects signed an informed consent prior to participating in this study.

### 2.1. Participants

Seventy-one postlingually deaf adult patients with bilateral severe and (or) profound sensorineural hearing loss participated in this study; they were implanted at the Cochlear Implant Department of the First Affiliated Hospital of Anhui Medical University, Anhui, China, from January 2016 to December 2020. Baseline information was collected before activation of the cochlear implant processor. The demographic data contained gender, duration of wearing HA before implant, age at implant, duration of CI use, and the results of self-assessment at the last visit.

### 2.2. Measurements

Data were collected via a voluntary online questionnaire.

The measurement used to assess the HRQOL of patients is HUI3. HUI3 is a self-completing questionnaire to evaluate health conditions from eight attributes, vision, hearing, speech, ambulation, dexterity, emotion, cognition, and pain; each dimension has five or six levels. Each level corresponds to a certain score which is used to be normalized to a utility from 0 to 1. 1 represents perfect health, and 0 represents the worst health. There are two ways to obtain the HUI3 scores single-attribute utility scores and multiattribute scores. Single-attribute utility scores were assessed when evaluated the changes of a single attribute. Multiattribute scores were used to compare integrated changes [6, 7].

RETRACTED

### 2.3. Data Analysis

The SPSSAU20.0 software was used for statistical analysis. Paired sample *t*-test was used to compare preoperative with postoperative scores. Multivariable linear regression was used to detect demographic variables associated with primary HUI3 multiattribute scores (preoperative HUI3 multiattribute scores) and gain in HUI3 multiattribute scores. Pearson's correlation tests were used to discover relationships among attributes that had statistically significant differences before and after CI.

## 3. Results

Table 1 shows the detailed demographic data of gender, age at implant, the time of hearing aid (HA) use before CI surgery, education level, residential settings, and duration of CI use. There were 44 women and 27 men; the mean age at implant was 32 years (SD, 10.56.5; range, 18 to 62 years). The median time of HA use before surgery was 4 years (p25, p75, 0,13; range, 0 to 37 years). Mean duration of CI use was 28.73 months (SD, 18.78; range, 6 to 65 months)

HUI3 single-attribute scores and multiattribute scores were obtained from 71 participants. As shown in Table 2, the HUI3 multiattribute scores and four HUI3 single-attribute scores including hearing, speech, emotion, and pain were statistically changed before and after the operation, and the difference between before and after the operation was statistically significant. The change in hearing and emotion was the most obvious among two of these four attributes, which may be related to the lower preoperative score.

Table 3 shows the multivariable linear regression result that the factors associated with preoperative HUI3 multiattribute scores and gain in HUI3 multiattribute scores. For preoperative HUI3 multiattribute scores, being female (vs male) and higher level of education (vs primary and below) were associated with better HUI3 scores before CI. The length of HA used before CI, the duration of CI use, stimulation condition, and the age at operation had no impact on the gain in HUI3 multiattribute scores. Primary hearing and emotion state were found to be significantly associated with the gain in HUI3 scores after CI.

RETRACTED

Pearson's correlation analysis shows the correlation between the change in the four attributes. There was a statistically significant positive correlation between change in hearing and change in emotion. Although the correlation between the change in hearing scores and change in pain scores was not significantly correlated, there was a statistically significant positive correlation for change in pain when compared to the change of emotion, as shown in Table 4.

The result showed no statistically significant difference for change in hearing scores in relation to the alteration of speech scores, and in this study (as shown in Table 4), 42.25% adults reached the best level of speech before CI. When we further divided patients into two groups according to whether having speech change caused by CI, the group with speech change had better hearing scores than those without speech change after CI (as shown in Table 5).

## 4. Discussion

In this study, we analyzed the HUI3 scores after bilateral or unilateral cochlear implant of a group of 71 adults with postlingual sensorineural hearing loss and detected the factors influencing the change.

In this cohort, preoperational HUI3 scores were around 0.31, and it had grown to about 0.70 after implant, and the quality of life had been greatly improved. For preoperative HUI3 multiattribute scores, being female and having a higher education level would have a better quality of life. Sousa's research reported the same result that the level of education is correlated with the quality of life using the WHOQOL-BREF questionnaire [2]. Other demographic varieties such as the residential settings, and the length of HA use, had no effect on the quality of life preoperatively. Concerning the gain in HUI3 multiattribute scores, the duration of HA use and the age at CI had no impact on the gain of HUI3 scores, which means that if other conditions are same, patients with different ages at implant would obtain the same improvement of quality of life. As for the time of CI use, other researches found that HUI3 scores change at the first year after implant, and then, the change is not obvious after that [8]. In these articles, HUI3 was firstly evaluated in the first year after CI. In this study, the follow-up time was from 6 to 65 months, showing there was no statistically significant correlation with the gain of HUI3 scores. Therefore, what is the exact time HUI3 scores improve is not sure.

In keeping with Müller, who reported that those patients with worse hearing levels before surgery were more likely to gain more HUI3 scores after CI [6], the regression analysis illustrated that primary hearing level had a large impact on the gain in quality of life. It reflected that the population with poorer hearing may achieve higher health quality postoperatively. The association we found between baseline emotion state and change in the quality of life significantly proved that emotional state is an important factor to influence the quality of life in qualified patients with hearing loss. The primary emotion score was also a contributor to the improvement of quality of life. We found the worse the emotion status preoperatively the more gain for the patient in quality of life.

RETRACTED

Multivariable linear regression showed that the stimulation condition (bilateral or unilateral) would not affect the quality of life, which is similar to Ramakers [4] and Sousa's reports [2]. Deaf adults have difficulties in social life, which could suffer from anxiety and depressive stress. Studies have proven that the intervention of CI was not only improving the HUI3 hearing level but also promoting other attribution levels. Mo et al used a generic measure, the SF-36, and found one scale, general health statistically significant different after CI [9]. Christoph et al had performed a prospective study which showed that the SF-36 scores improvement was statistically significant in two domains, mental health and social functioning [5]. Louise et al detected that three HUI3 subdomains of hearing, emotion, and speech significantly improved because of CI [10]. Hanna et al reported that patient only hearing and speech scores improved significantly according to HUI3 measurement after CI [11]. Summerfield's study reported great change in hearing and speech using HUI3 and a difference in depression using EQ-5D-3L [12]. Therefore, using different measurements would find different dimensions of change in the quality of life. Even performing the same measurement could get different results. A possible explanation might be the difference of the evaluated subjects' living environment, social form, or life style. In our study, the scores were significantly improved in four domains, hearing, speech, emotion, and pain. Adolescents with hearing loss could feel isolated, embarrassed, and depressive [13], and we hypothesis that the change of emotion after CI was associated with the hearing improvement, and when patients' hearing ability improved, the depressive emotion could be changed accordingly. In this study, we confirm this hypothesis, the more change in hearing after CI, the better emotion changed. Apart from that, the attribution of speech and pain were also significantly improved postoperatively. Is there existing a relationship among changes in these dimensions? Pearson analysis shows that the change of HUI3 speech has no relation with the variation of hearing. Possibly because, almost 42.25% of subjects reached the best speech level preoperatively. Therefore, we divided patients into two groups according to speech change, and the postoperative hearing scores of patients with speech change were significantly better than those without speech change. This means the hearing level after CI could influence the verbal expression ability of the patient.

RETRACTED

The pain score of our patients was raised as well due to CI. Pearson correlation analysis showed the change of the pain scores had no relation with hearing improvement. If hearing improvement was not the direct cause of change in HUI3 pain scores, what was the reason for pain perception improvement after CI? The pain and emotion are converged on the anterior cingulate and insular cortices [14]. It is testified that a hybrid emotion-focused remedies may be an available intervention for chronic pain patients with comorbid emotional problems. Emotion regulation may be one factor of pain development and maintenance [15, 16]. Therefore, we hypothesis that there was a correlation between the change of pain and the improvement of emotion postoperatively. It is not surprising to discover outcomes of the pain scores had a statistically significant correlation with the gain in emotion. This indicates CI improved hearing levels, which then raised emotion level and finally positively influence on pain perspective.

The present study identified CI had effectively improved hearing, speech, emotion, and pain, which made statistically significant improvement in quality of life among postlingually deaf adults. There was a statistically significant association between the change of emotion state and improvement in hearing level. We also found a statistically significant correlation between the reduction of feeling in pain and improvement in emotion state. Sex and education level significantly influence the quality of life preoperative. Duration of HA use, age at implant, time of CI use, and bilateral or unilateral did not significantly impact the improvement in quality of life. The change of quality of life seemed to be influenced by the primary state of emotion and hearing. The HUI3 measure is suitable for this cohort of patients.

## Figures and Tables

**Table 1:** Demographic data of 71 adults.

	*N*	%
Gender		
Male	27	38.03
Female	44	61.97
Age at CI (yrs)		
18–30	35	49.30
31–40	22	30.99
41–62	14	19.71
Length of HA use (yrs)		
0–1	29	40.85
2–10	22	30.99
11–32	20	28.16
Educational status		
Primary	13	18.31
Middle and high school	34	47.89
University and above	24	33.80
Residential setting		
Urban	35	49.30
rural	29	40.84
suburban	7	9.86
CI implant side		
Bilateral	19	26.76
Unilateral	52	73.24
Time of CI use (mos)		
6–12	25	35.21
13–36	20	28.17
37–65	26	36.62

RETRACTED

**Table 2:** HUI3 multiattribute scores and four HUI3 single-attribute scores pre- and post-CI.

	Pre-CI	Post-CI	Gain	*t*	*p*
HUI3 multiattribute	0.32 ± 0.26	0.70 ± 0.22	−0.38	−13.404	0.000^*∗∗∗*^
HUI3 hearing	0.24 ± 0.27	0.72 ± 0.24	−0.48	−15.731	0.000^*∗∗∗*^
HUI3 speech	0.77 ± 0.29	0.85 ± 0.26	−0.08	−5.207	0.000^*∗∗∗*^
HUI3 emotion	0.66 ± 0.36	0.93 ± 0.16	−0.28	−6.255	0.000^*∗∗∗*^
HUI3 pain	0.93 ± 0.19	0.99 ± 0.02	−0.06	−2.792	0.007^*∗∗*^

All scores show as mean ± SD. ^*∗*^*p* < 0.05; ^*∗∗*^*p* < 0.01; ^*∗∗∗*^*p* < 0.001.

**Table 3:** Factors associated with primary HUI3 scores and gain in HUI3 scores.

Variables		Primary HUI3 scores (*n* = 71)					Gain in HUI3 scores(*n* = 71)				
		*B*	95% CI	*T*	*p*	VIF	B	95% CI	*t*	*p*	VIF
Gender	Male	—	—	—	—	—	—	—	—	—	—
	Female	0.149	0.012–0.286	2.13	0.037^*∗*^	1.409	—	—	—	—	—
Education status	Primary and below	—	—	—	—	—	—	—	—	—	—
	Middle and high school	0.228	0.057～0.398	2.618	0.011^*∗*^	2.306	—	—	—	—	—
	University and above	0.248	0.084～0.483	2.784	0.007^*∗∗*^	2.835	—	—	—	—	—
Residential setting	Rural	—	—	—	—	—	—	—	—	—	—
	Urban	−0.002	−0.153～0.148	−0.032	0.975	1.796	—	—	—	—	—
	Suburban	0.004	−0.199～0.206	0.035	0.972	1.157	—	—	—	—	—
Time of HA use before CI		−0.003	−0.011～0.005	−0.740	0.462	1.392	0.000	−0.005～0.006	0.159	0.874	1.254
Age at CI		−0.004	−0.010～0.002	−1.299	0.199	1.313	0.002	−0.002～0.007	0.921	0.361	1.576
Stimulation condition	Unilateral	—	—	—	—	—	—	—	—	—	—
	Bilateral	—	—	—	—	—	−0.022	−0.119～0.076	−0.430	0.668	1.312
Time of CI use		—	—	—	—	—	0.000	−0.002～0.003	0.296	0.768	1.162
Primary HUI3 hearing		—	—	—	—	—	−0.470	−0.879～−0.062	−2.257	0.028^*∗*^	1.273
Primary HUI3 emotion		—	—	—	—	—	−0.762	−0.983～−0.541	−6.756	0.000^*∗∗∗*^	1.293
Primary HUI3 speech		—	—	—	—	—	0.394	−0.075～0.863	1.645	0.105	1.276
Primary HUI3 pain		—	—	—	—	—	−0.377	−0.909～0.156	−1.378	0.107	1.372

^*∗*^ *p* < 0.05; ^*∗∗*^*p* < 0.01; ^*∗∗∗*^*p* < 0.001.

**Table 4:** Correlation coefficient between gain of HUI3 four attributions.

	Change in HUI3 hearing *r*(*p*)	Change in HUI3 speech *r*(*p*)	Change in HUI3 emotion *r*(*p*)	Change in HUI3 pain *r*(*p*)
Change in HUI3 hearing	—	0.039(0.7459)	0.336(0.004^*∗∗*^)	0.087(0.470)
Change in HUI3 speech	—	—	0.088(0.464)	−0.006(0.959)
Change in HUI3 emotion	—	—	—	0.248(0.037^*∗*^)
Change in HUI3 pain	—	—	—	

*r*, correlation coefficient; *p* (*p* value), statistically significant result. ^*∗*^*p* < 0.05; ^*∗∗*^*p* < 0.01; ^*∗∗∗*^*p* < 0.001.

**Table 5:** The HUI3 hearing scores of the groups with or without speech change after CI.

	Groups (mean ± SD)		*t*	*p*
	Group without speech change	Group with speech change		
HUI3 hearing scores	0.67 ± 0.26	0.81 ± 0.17	−2.747	0.008^*∗∗*^

^*∗*^ *p* < 0.05; ^*∗∗*^*p* < 0.01.

RETRACTED

## Data Availability

The simulation experiment data used to support the findings of this study are available from the corresponding author upon request.
